The article "Research on the Integration and Development of Ecotourism Industry and Sports Health Industry under the Background of Rural Revitalization Strategy" was retracted in 2023. Reasons: unreliable results or conclusions; concerns about the data; concerns about the peer review; concerns about the citations.

# Research on the Integration and Development of Ecotourism Industry and Sports Health Industry under the Background of Rural Revitalization Strategy

**DOI:** 10.1155/2022/3343297

**Published:** 2022-02-11

**Authors:** Xiaoxiao Zhao

**Affiliations:** Henan Institute of Economics and Trade, Zhengzhou, Henan 450000, China

## Abstract

With the growth of people's consumption demand and the popularization of transportation, ecotourism has gradually entered people's vision and become a fashionable choice for people's leisure. Since the reform and opening up, tourism has increasingly become a popular and popular form of consumption. It appears in people's life and has the characteristics of personalization, leisure, and diversification. Based on the understanding of the current situation of the integrated development of ecotourism and sports tourism, this paper discusses the integrated development strategy of the ecotourism industry and sports health industry. As an important content and component of rural industry, it is very necessary to promote the better development of ecotourism. It is also an important task to implement the Rural Revitalization Strategy. It has important value and significance for improving the rural industrial structure and promoting rural economic development. The purpose of this study is to promote the coordinated development of the ecotourism and sports health industry and to provide help for the stable development of tourism in the market competition environment.

## 1. Introduction

With the rapid development of tourism and the increasing demand for tourism, in recent years, ecotourism has attracted a large number of sports lovers with its simple rural environment and beautiful natural landscape [1]. Ecotourism is an industry with farmers as the main body, rural folk culture as the core, and urban residents as the main target customers. The purpose of developing ecotourism is to lead farmers to get rich and promote rural economic development [2]. The integration of ecotourism and sports tourism breaks the traditional single agritainment tourism mode. By combining the open ecotourism resources with sports tourism, it can enrich the tourism content and realize people's life pursuit of cultivating sentiment and strengthening body [3]. In addition to the extensive use of the Online Intelligent Tourism platform, the traditional single ornamental tourism project is gradually replaced by experiential tourism, that is, consumers intuitively perceive and experience culture and atmosphere in the process of tourism [4]. As an important content and component of rural industry, ecotourism is very necessary to promote the better development of ecotourism, which is also an important task in the implementation of Rural Revitalization Strategy and has important value and significance in the improvement of rural industrial structure and rural economic development [5].

Since the reform and opening up, tourism has increasingly become a popular and popular form of consumption, appearing in people's lives, and showing the characteristics of personalization, leisure, and diversification [6]. With the growth of people's consumption demand and the popularity of transportation, ecotourism has gradually entered people's vision and become a fashion choice for leisure [7]. In order to break the urban-rural dual structure and promote the integrated development of urban and rural areas, the Party Central Committee timely put forward the “Rural Revitalization Strategy,” which aims to lead the direction of rural reform and development in the new era, comprehensively stimulate the vitality of rural development, and establish and improve the system and mechanism to accelerate the sustainable development of rural economy and society [8]. Rural sports tourism is based on the natural and cultural environment resources in rural areas to meet the tourists' health and entertainment through sports activities [9]. The development of rural sports tourism is conducive to balancing the relationship between urban and rural areas, adjusting the rural industrial structure, promoting rural economic development, and achieving the goal of national fitness and national health [10]. Based on the current situation of the integration development of ecotourism and sports tourism, this paper discusses the integration development strategy of the ecotourism industry and sports health industry, aiming to promote the coordinated development of ecotourism and sports tourism and provide help for the stable development of the tourism industry in the market competition environment.

## 2. Problems in the Development of Sports Tourism and Ecological Tourism

### 2.1. Tourism Project Development Project Is Too Single

The connotation of sports tourism and rural sports tourism: sports tourism is the integration and intersection of sports and tourism. It reflects the sociality of sports and tourism. Sports tourism is not only an industrial branch of social sports but also an important part of tourism. It is a kind of special tourism and new tourism activity in human social life. Its concept can be divided into broad and narrow senses.

Sports tourism and ecotourism development model are very similar, but in the process of development, local unique ecotourism and sports tourism resources are not excavated from local characteristics, which makes sports tourism and ecotourism complex projects single, and tourism integration development lacks necessary facilities and equipment support. In the process of integration and development of ecotourism and sports tourism, it is necessary to deal with the relationship between services and consumers, which affects the implementation effect of tourism projects and the sustainability of the overall industry development. Under the influence of rural revitalization, ecotourism has also made many achievements, but there are still many problems. They do not have a complete and unified plan, which basically belongs to decentralized development, no unified layout, and no clear subject of tourism projects.

From the questionnaire of 300 people randomly on the website, we can get the data of distress reasons when arranging trips, which can be used as one of the references of demand analysis. The data are shown in Table 1.

Under the action of rural revitalization strategy, the demand of Chinese residents for rural sports tourism is increasing, but the types of tourism products in the tourism market cannot meet the growing demand of people, which reduces the expectation of consumers for rural sports tourism products and hinders the sustainable development of tourism industry in the new environment. The reason for this situation is that when developing brand-new tourism projects, most areas put too much energy into optimizing construction in order to obtain more economic profits [11]. In the development of sports tourism and ecotourism in some places, some people do not know enough about the protection policies and related knowledge of intangible cultural heritage in the field of sports and even do not have some scientific protection consciousness, which leads to the loss of intangible cultural heritage resources that local sports tourism and ecotourism depend on. In the process of integration of sports tourism and ecotourism, some people lack understanding of the protection policy of intangible cultural heritage in the sports field and even lack scientific protection consciousness in the process of tourism, which leads to the increasingly serious loss of intangible cultural heritage on which sports tourism and ecotourism depend.

### 2.2. Rural Cultural Ecology Gradually Disappeared

With the accelerating pace of life, most urban residents are eager to relieve stress by changing the environment and enriching their life after work. In this context, ecotourism and sports tourism industries are gradually emerging, and some developers face the regional advantages of rich tourism resources, hoping to take ecotourism development as a breakthrough point to enhance economic benefits, and then cause a boom in tourism development in rural areas. Ecotourism wants to develop healthily, and there is a great demand for professionals. However, the current situation is that the demand for talents is not directly proportional to the training of talents. There is no unified, professional, and systematic training institution in the training of professional personnel. The employees are basically local people, and the professional training does not go deep into the countryside, resulting in the low quality of tourism professionals. Ecotourism is more of a spiritual tourism experience, which enables urban residents to understand local customs in different ecological environments and gain deep cultural feelings. However, some developers neglect the protection of the ecological environment, and even transform some ecological resources in a subjective way, providing modern leisure places for urban residents, which makes ecotourism development lose its original meaning.  Figure 1 shows the general law of rural development.

Ecotourism is actually a kind of experience tourism and a kind of sports tourism. This kind of tourism makes tourists from cities get a more personal feeling of rural culture in the process of experiencing local customs. However, the farmers who run the business excessively pursue how to meet the needs of urban tourists and even arbitrarily transform the ecotourism resources with local characteristics into leisure venues that adhere to the taste of urban life, thus making some ecotourism and sports tourism development go the other way and lose the foundation of sustainable development [12]. Driven by the integration of sports tourism, ecotourism and farmers' desire to get rich, farmers raise funds to set up tourism in some areas with rich ecotourism resources. In the process of setting up rural sports tourism, farmers destroyed the rural cultural-ecological environment and even artificially transformed the ecotourism resources with local characteristics into leisure venues with the taste of vassal cities, which made the development difference between ecotourism and sports tourism increase.

## 3. The Combination of Sports Tourism and Ecological Tourism

### 3.1. Strengthen the Interaction between Sports Health Industry and Ecotourism

For better development of ecotourism, more development space must be developed. As the core of tourism development, rural culture is an important part of Chinese culture. This is a good development direction. Therefore, it is necessary to combine local natural conditions and resource characteristics, according to market demand, focus on promoting characteristic culture and geographical advantages, innovate some colorful and distinctive cultural tourism products, and give play to the unique advantages of rural ecology and cultural resources. In the process of the integration of ecotourism and sports tourism, government departments can issue a series of policies to encourage people to realize the effective use of ecotourism resources and encourage local college students to use their spare time in rural development areas through appropriate preferential policies. Carrying out survival training in the wild or carrying out extracurricular sports constantly attracts more rural sports tourism participants to participate.

The added value of the sports industry is defined as the *X*_0_ series, and the other sports industries are defined as the *X*_i_ series. Then, the data is initialized, that is, the *X*_0_ sequence is divided by the *X*_i_ sequence, and the original data is nondimensionalized. The sequence was put into the following formula to get the average correlation coefficient *L*_0*i*_(*k*):

(1) $$\begin{array}{c} L_{0i}\left(k\right)=\frac{\left(\min|X_{0}\left(k\right)-X_{i}\left(k\right)|+\rho \max\left|X_{0}\left(k\right)-X_{i}\left(k\right)\right|\right)}{\left(|X_{0}\left(k\right)-X_{i}\left(k\right)|+\rho \max\left|X_{0}\left(k\right)-X_{i}\left(k\right)\right|\right)}. \end{array}$$

In the formula, *ρ* is the resolution coefficient, *ρ* ∈ (0, 1), and generally, *ρ* = 0.5. *L*_0*i*_ (*k*) is the average correlation coefficient, which means the average correlation between the added value of each major sports industry and the added value of China's sports industry. The correlation degree calculation is solved by the mean value method, *i* is each sports industry, *k* is the year, let the correlation degree of sports industry *i* to the total output value of the reference sequence 0 be *G* (0, 1), and *n* is the number of correlation coefficients of the comparison sequence, which is

(2) $$\begin{array}{c} G\left(0,1\right)=\frac{1}{n\sum_{k=1}^{n}L_{0i}\left(k\right)}. \end{array}$$

In the process of tourism projects and resource development, the relevant personnel should examine the existing problems in the past with a development perspective and explore innovative development ways to provide guidance for resource development with new ideas [13].  Figure 2 shows the contribution of different resources in different rural development stages.

Driven by the rural revitalization strategy, we can make better use of rural characteristics to establish new tourism projects and strive to develop leisure agriculture so that tourists can integrate sightseeing, picking, and experiencing farming activities in the process of playing. In this way, they will meet their needs of understanding farmers' lives and enjoying local tastes better. Besides, they also need to build corresponding accommodation and vacation projects. At the same time, it is necessary to coordinate the relationship between people, consider the fairness of benefit distribution from different angles, avoid damaging the ecological environment, expand people's communication and development space, and realize the harmonious development of people. The interactive development of sports tourism and ecotourism should be based on folk sports characteristics, combine with the needs of market development, fully integrate natural ecotourism, rural cultural tourism, and rural sports tourism resources, create a point-line-plane-integrated tourism pattern, scientifically position and develop sports health industry products according to the development needs of sports tourism and ecotourism, and create an interactive development mechanism of sports health industry and ecotourism with distinctive local characteristics.

### 3.2. Vigorously Develop Ecological Tourism

Ecotourism projects include landscape agriculture projects. The development of this tourism direction reflects the constant innovation of ecotourism. The main purpose of this project is to preserve the agricultural experience, develop on the basis of rural scenery, and design and build a landscape with rural characteristics so as to make ecotourism more distinctive. In the process of the combined development of ecotourism and sports tourism, aiming at the problem of destroying the ecological environment, we should take ecological resources protection as the main idea and deeply discuss the countermeasures for the integration and development of the two and the ways of resource development. According to the rural revitalization strategy, ecotourism products will be continuously increased, new formats with rural characteristics will be created, ecotourism destinations and boutique tourism routes will be created according to different themes, folk customs and health bases with rural characteristics will be built, different tourism products will be provided, and more new services will be added. The rapid development of network technology has expanded the scope of media communication. As a new tourism industry, the integration of ecotourism and sports tourism should not only strengthen the connotation construction but also make use of modern media resources to increase the publicity of tourism projects so that more people can understand the characteristics of rural sports tourism and participate in tourism projects, thus creating more benefits for industrial development.

## 4. Conclusions

Today, with the increasing demand for tourism services, the integration and development of ecotourism and sports tourism have become an inevitable development trend. Both of them have inherent cultural spirit in the process of development, and this culture is also the basis of their integration, development, and utilization. As a new tourism industry, the integration of rural sports tourism and sports tourism plays an important role in promoting urban-rural integration and industrial innovation. The development of ecotourism and sports tourism must have its own cultural connotation, which is the potential characteristic of its development and the premise of its sustainable development. In order to realize the coordinated development of the two, it is necessary to highlight the characteristics and advantages of ecotourism and sports tourism, realize the steady growth of the number of tourists, and create a more orderly market environment for the industry by rationally allocating resources and optimizing tourism services. To develop ecotourism under the background of rural revitalization strategy, it is necessary to fully combine the natural scenery, characteristic culture, and characteristic crops in the countryside, enrich the ecotourism content, and realize the sightseeing value and cultural dissemination value of ecotourism.

## Figures and Tables

**Figure 1:** The general law of rural development.

**Figure 2:** The contribution of different resources in the development stage of the tourism economy.

**Table 1:** Data of distress reasons during trip arrangement.

Cause	Dining arrangements	Accommodation arrangements	Traffic safety	Opening hours of scenic spots
Number	32	121	111	36
Proportion (%)	10.7	40.3	37.0	12.0

## Data Availability

The data used to support the findings of this study are included within the article.
